The article "An Intelligent Analysis System for Traditional Arts and Crafts Based on Digital technology: Taking the Guangdong-Hong Kong-Macao Greater Bay Area as the Observation Center" was published in 2022. Journal: Comput Intell Neurosci.

# An Intelligent Analysis System for Traditional Arts and Crafts Based on Digital technology: Taking the Guangdong-Hong Kong-Macao Greater Bay Area as the Observation Center

**DOI:** 10.1155/2022/5799198

**Published:** 2022-04-25

**Authors:** Tingting Wen, Sijie Fan

**Affiliations:** ^1^Rao Zongyi Cultural Research Institute of Shenzhen University, Shenzhen 518000, China; ^2^School of Fine Arts and Design, Guangzhou University, Guangzhou 510000, China

## Abstract

In order to improve the analysis effect of traditional arts and crafts, this paper analyzes traditional arts and crafts combined with digital technology, builds an intelligent analysis system to improve the digital processing effect of traditional arts and crafts, and takes the Guangdong-Hong Kong-Macao Greater Bay Area as an example to verify the system effect. In order to improve the accuracy of subsequent image alignment and defect detection, this paper compares the effects of the pixel-level edge detection algorithm and the subpixel-level edge detection algorithm and finally selects the subpixel-based edge detection algorithm to extract the edge of the image. In addition, this paper compares the traditional defect detection algorithm through research and experiment and proposes an improved image phase difference method according to the actual situation. The experimental research shows that the traditional arts and crafts intelligent analysis system based on digital technology proposed in this paper has a very good effect. At the same time, with the support of this system, the intelligent analysis of traditional arts and crafts in the Guangdong-Hong Kong-Macao Greater Bay Area can be carried out efficiently.

## 1. Introduction

With the development of new technologies and the evolution of media forms, the forms of emerging media in assisting the inheritance of traditional arts and crafts are becoming more and more diverse and comprehensive. Moreover, it is obviously interdisciplinary and intradisciplinary, and it faces a wide range of audiences from path innovation to countermeasures, and its research boundaries continue to expand [1]. The new media assistance method is more targeted and adaptable in matching and integrating with the content of traditional arts and crafts, which provides more possibilities for the inheritance and development of traditional arts and crafts. However, in general, there are still some problems in the related research. From the perspective of theoretical research, some literature have weak theoretical foundations or even not cited, and the research still remains at the level of specific methodology. With various changes in the field of new media, related research needs to introduce and learn from theoretical resources to make up for the theoretical gap and enhance the persuasiveness of the research [2]. From the perspective of practical operation research, different traditional arts and crafts categories have different inheritance and dissemination types, and the content dimensions are wide. However, the research on inheritance methods and dissemination methods is mainly aimed at the macroscopic content and external characteristics of traditional arts and crafts, and there is no systematic research on specific categories [3].

The development of Chinese traditional arts and crafts is national and regional and occupies a very important position in the development of traditional culture. Introducing traditional arts and crafts into modern graphic design can change the design concept and promote the update of related design concepts, which can not only highlight the characteristics in the design but also promote the innovation of traditional arts and crafts. The most important thing in modern graphic design is the application of traditional arts and crafts and the expression of aesthetic cognition. Therefore, traditional arts and crafts can have a place in modern graphic design.

The effective inheritance of traditional arts and crafts in contemporary society needs to be achieved through efficient communication, and the communication needs to rely on the carrier power of media. Therefore, using new media to spread traditional arts and crafts can promote the inheritance and development of traditional arts and crafts in contemporary society. Propagation refers to the diffusion and transmission of information, and activities such as information transmission, reception, and feedback are realized with the help of meaningful symbols. For the dissemination of traditional arts and crafts, it is necessary to protect and inherit. Traditional arts and crafts are the core content of dissemination, the carrier of dissemination is specific artwork, and the form of dissemination corresponds to the process of making, viewing, using, and displaying products. Therefore, the means of dissemination of traditional arts and crafts have diverse characteristics, among which new media is the means that needs to be mainly utilized in the dissemination of contemporary traditional arts and crafts. The dissemination of traditional arts and crafts using new media as a carrier can shorten the distance between people and traditional arts and crafts, enhance people's awareness and sense of responsibility for inheriting and developing traditional arts and crafts, and promote the effective inheritance of traditional arts and crafts in contemporary society.

This paper analyzes traditional arts and crafts combined with digital technology, builds an intelligent analysis system, improves the digital processing effect of traditional arts and crafts, and takes the Guangdong-Hong Kong-Macao Greater Bay Area as an example to verify the system effect.

## 2. Related Work

McCartney and Tynan [4] proposed that national culture is the soul and foundation of a nation, and the protection of “intangible cultural heritage” should adhere to the principle of overall protection. Lockheart [5] analyzes local governments' efforts in the protection and utilization of “intangible cultural heritage” from nine aspects, including policy formulation, value maintenance, win-win cooperation, social coordination, functional integration, performance evaluation, task implementation, informatization construction, and resource mobilization. The specific role positioning has been explored in depth. Sachdev [6] proposes that when museums play the role of heritage inheritance, they should take “hierarchical” protection measures; Andreeva et al. [7] believe that no matter what kind of protection, the law is the foundation. Nebessayeva et al. [8] pointed out that legal protection of “intangible cultural heritage” is a consensus reached by the theoretical and practical circles, and analyzed how legal means can play the role of protecting “intangible cultural heritage” from three aspects: value target positioning, legislative guiding ideology, and integration of legal norms actual effect. Mourtzis [9] proposes that in order to realize the protection of “intangible cultural heritage” in the true sense, we should start from the protection of the cultural space on which the heritage depends for survival and inheritance. Klockars et al. [10] believe that foreign cultural erosion is an important factor in destroying “intangible cultural heritage.” The traditional protection methods, whether recording “intangible cultural heritage” through audio, text, video, and so on, or subsidizing inheritors to stimulate inheritance, are all temporary solutions. Without curing the root cause, the effective protection of “intangible cultural heritage” must satisfy sustainability, adapt to the dynamism of the development of the times, be able to arouse the emotional resonance of the audience, and be able to achieve certain utilitarian purposes in the practice of “intangible cultural heritage.”

Hermus et al. [11] proposed that the protection of traditional handicrafts should not be limited to economic cognition and economic value expectations, but should be protected and developed from the rich social meaning of manual production methods. Calvert and Schyfter [12] believe that the productive protection of craftsmanship Danqing in northern Shaanxi is not successful and takes this as an example to illustrate that in order to promote the inherent culture of traditional handicrafts, it should enter the modern knowledge system and be understood and accepted by contemporary society in order to achieve its effective protection. Greene et al. [13] pointed out that the productive protection of traditional handicraft skills should respect the “core skills,” and through prudent innovation of technology, brand creation, introduction of talents, and strengthening of marketing, and so on, so that the ancient skills can continue to form productivity in the contemporary era is the inherent protection and development of skills. The best way of human value. Liu et al. [14] mentioned that in the process of developing the handicraft industry, the emergence of contradictions is inevitable, and the relevant functional departments of the government should assume the responsibility of research, demonstration, and scientific analysis to ensure effective scientific development. Luo and Dai [15] deeply analyze the productive protection of paper-cutting and propose that traditional handicrafts, such as paper-cutting and other “intangible cultural heritage,” can be integrated into contemporary production practices in new forms and ways to gain space for continued existence. On one hand, the academic circles have recognized the positive role of productive protection in the protection of traditional handicrafts. On the other hand, they have also begun to worry about the problems that may arise in productive protection. Knight et al. [16] believes that productive protection should avoid over-exploitation and prevent the commercialization, industrialization, and tourism of heritage resources. Jordan and O'Donoghue [17] propose that large-scale mechanical production must not completely replace manual work, resulting in destructive development but also believe that the productive protection of traditional handicrafts cannot completely avoid commercialization and industrialization. In summary, productive protection is an important way to protect traditional handicrafts, and industrialization, as one of the important modes of productive protection, is regarded as a “flood beast” by many scholars, equating industrialization with the repeated production of large machinery, out of protection. The original intention of “intangible cultural heritage” traditional handicrafts has adopted an attitude of refusal to industrialization. But in fact, industrialization is only a method and means, as long as the principle of protecting core skills and cultural connotations is adhered to, industrialization can instead promote the protection of traditional crafts [18].

For traditional handicrafts “intangible cultural heritage” projects, without screening whether they are suitable for industrial development, blindly and wishful thinking will have the opposite effect, not only will it fail to protect the inheritance, but will it will cause irreversible damage to the “intangible cultural heritage” project itself [19]. Therefore, whether traditional handicraft projects can be industrialized and how to be industrialized need to be considered and treated differently and cannot be generalized. Just as Yue Qing's point of view: developing “intangible cultural heritage” into a cultural industry is not the only and necessary way for productive protection.

## 3. Digital Art Image Processing

The first step of image preprocessing is to deal with the noise in the image. There are mainly three types of noise in the image: additive noise with a normal distribution, multiplicative noise caused by the CCD movement during photoelectric conversion, and salt and pepper noise caused by the amplifier. If the original image is *f*(*x*, *y*) and the image with noise is *f*′(*x*, *y*), there are:

(1)   Additive noise: The additive *n*(*x*, *y*) histogram approximately obeys the normal distribution, and then there are
  (1) $$\begin{array}{c} f^{\prime }\left(x,y\right)=f\left(x,y\right)+n\left(x,y\right). \end{array}$$
(2) Multiplicative noise: We assume that the multiplicative noise is *χ*(*x*, *y*), where *χ*(*x*, *y*) may approximately obey the normal distribution, uniform distribution, exponential distribution, and so on, and then there are
  (2) $$\begin{array}{c} f^{\prime }\left(x,y\right)=f\left(x,y\right)\times \chi \left(x,y\right). \end{array}$$
(3)   Salt and pepper noise: Salt and pepper noise is ordinary black and white dots, and its expression is as follows:
  (3) $$\begin{array}{c} f^{\prime }\left(x,y\right)=\left\{\begin{array}{cc} 0, & f\left(x,y\right)<d,\\ 255, & d\leq f\left(x,y\right)\leq 2d,\\ f\left(x,y\right), & \text{other.} \end{array}\right. \end{array}$$
For these noises, typical spatial domain filtering methods include Gaussian filtering, mean filtering, median filtering, and so on.

Owing to the particularity of the detection requirements of this subject, the selection of the smooth function should take into account the removal of salt and pepper noise without affecting the defect detection. Therefore, the image smoothing algorithm used in this paper is median filtering. The advantage of median filtering makes it possible to remove some isolated salt and pepper noise on the premise of preserving the edge of interest in the image. The principle of median filtering is to select the median value of the selected window pixels as the current pixel value. The one-dimensional mathematical expression of the median filter is as follows [20]:

(4) $$\begin{array}{c} f_{k}=\text{Middle}\left\{f_{x-n},f_{x-n+1},\cdots ,f_{k},f_{k+n-1},f_{\text{k}+n}\right\}. \end{array}$$

Among them, *f*_*k*_ is the gray value of the *k*th pixel of the image and Middle represents the median operation of the array. Here, there are (2*n* + 1) pixel gray values in the selected kernel window. The median filter is to output the median value of the gray values of all pixels in the sliding kernel window of the selected kernel window in the original image. According to actual needs, nuclear windows of different shapes and sizes can be selected, such as circular and square, and sizes such as (3 × 3), (5 × 5), and (7 × 7).

The size of the original image is *M* × *N*, and the size of the kernel window is (2*n* + 1) × (2*n* + 1).

For the detection image of this paper, except for some high-frequency edge parts of the image, most of the image background areas have similar gray values, and these areas are usually connected areas. According to the characteristics of the regional correlation of the image, this paper proposes a fast median filtering algorithm. When processing an image using the kernel window function, the sliding window function only moves one pixel horizontally or vertically, that is, a column or row of pixel values is added to the right or lower side of the window, and a column or row of pixel values is removed from the left or upper side. Therefore, for the median value of the current window, it is only necessary to consider the influence of the pixel values of the two columns or rows added and removed on the median value of the previous window. Therefore, the comparison of unchanged pixel values can be skipped, thus greatly reducing the time-consuming of the algorithm. Taking horizontal movement as an example, the specific steps are as follows:

1. The algorithm judges whether the pixel values corresponding to the row added to the column and the row removed from the column before and after the move are equal one by one. If they are equal, according to the characteristics of the correlation of pixel values of adjacent pixels, the value in this window remains unchanged, otherwise, the algorithm enters step (2). Since the background of the image to be detected in this paper accounts for 80% of the entire image, and the background is uniform, this step is the key to reducing time-consuming in this paper.
2. The algorithm defines and initializes a two-dimensional (2*n*+1) × (2*n*+1) window array and a one-dimensional 256 × 1 histogram array, and counts and saves the histogram in the window. However, in the saved histogram array, the value of the pixel value corresponding to the leftmost column of the previous window is subtracted by 1, and the value of the pixel value corresponding to the rightmost column of the current window is added by 1.
3. The algorithm accumulates the histogram array. When the accumulated value is equal to [(2*n*+1) × (2*n*+1)+1]/2, the pixel value on the corresponding histogram is the current median value.

We assume that the size of the kernel function is 3 × 3. The brief process of the improved fast median filter in this paper is shown in Figure 1 [21].

Among them, Figures 1(a) and 2(a) are the pixel values taken by the template when the original image slides, the yellow area on the left represents the pixel value before sliding, and the blue area on the right is the pixel value after sliding. Figures 1(b) and 2(b) are histogram array data tables. Figure 1 corresponds to the situation of step (1) above, and the median value before and after moving is 4. Since the background of the image of the product to be detected in the system is uniform and occupies most of the area of the image, the above step (1) can greatly reduce the time-consuming of the algorithm.  Figure 2 corresponds to the situation of steps (2) and (3), the median value is 4 before the template is moved, and the median value is 5 after the template is moved. We assume that the size of a kernel function is *N*=*n* × *n*. According to the data structure theory, it takes an average of *N*  log_2_  *N* comparisons to find the median value among *N* numbers. However, this paper only needs to compare $2\sqrt{N}$ times at most, and it will increase with the increase of the kernel function size.

Through a large number of experimental results, it is proved that the improved fast median filter algorithm in this paper not only guarantees the smoothing effect but also greatly reduces the time of image processing when the kernel function of the same size is used to smooth the image. In the whole comparison experiment, kernel functions of different sizes were selected, respectively, and the traditional median filter and the improved fast median filter algorithm in this paper were used to process the same size 240 × 656 image containing noise.

(5) $$\begin{array}{c} \text{MSE}=\frac{1}{M\times N}{\sum_{i=1}^{M}\sum_{j=1}^{N}\left[f\left(x,y\right)-g\left(x,y\right)\right]}^{2},\\ \text{PSNR}=20\log_{10}\left(\frac{255}{\sqrt{\text{MSE}}}\right). \end{array}$$

In the field of machine vision application systems, the contrast of images is often not high due to factors such as illumination. Therefore, it is necessary to purposefully extract image local features. In order to display the image features such as the region of interest and the edge of the original unclear image, it is necessary to enhance the image. The mathematical expression of the image enhancement algorithm in this paper is shown in formula (6):

(6) $$\begin{array}{c} g\left(x,y\right)=\text{round}\left(\left(f\left(x,y\right)-\text{mean}\right)*\text{Factor}+f\left(x,y\right)\right). \end{array}$$

Among them, *f*(*x*, *y*) is the original image, *g*(*x*, *y*) is the processed image, and round is the rounding operation, Factor is a coefficient, and mean is the gray value of the corresponding pixel after median filtering. The size of the kernel function selected in this paper is 17 × 17, and the Factor is 1.0.  Figure 3(a) is the original image, Figure 3(b) is the processing diagram of the histogram equalization algorithm, and Figure 3(c) is the processing diagram of the algorithm in this paper. It can be seen from the comparison diagram that this algorithm can well highlight the region of interest in the image.

The maximum between-class variance method is an efficient threshold segmentation method. This algorithm has been identified as the best algorithm among image threshold segmentation algorithms since its inception. Owing to the simple calculation process of the algorithm and the insensitivity to the brightness and contrast of the image, the algorithm has a wide range of applications. The image segmentation algorithm used in this paper is this algorithm. The algorithm works as follows:

For image I, *T* represents the value between the image background and foreground segmentation, the number of pixels occupied by foreground and background are *n*_0_ and *n*_1_, respectively, the average grayscale values of the background and foreground are *λ*_0_ and *λ*_1_, the mean is denoted as *μ*, and the interclass variance is denoted as *σ*^2^, there are:

(7) $$\begin{array}{c} \mu =n_{0}\lambda_{0}+n_{1}\lambda_{1},\\ \sigma^{2}=n_{0}{\left(\lambda_{0}-\mu \right)}^{2}+n_{1}{\left(\lambda_{1}-\mu \right)}^{2}. \end{array}$$

When this algorithm is used to traverse the entire image to obtain the maximum value of the interclass variance *σ*^2^, the value of *T* is the best threshold for segmentation. The effect of using the OTSU threshold on the enhanced detection area is shown in Figure 4. The algorithm can perfectly separate the detection area from the background.

The pixel-level edge contour extraction algorithm is as follows:

(1) *Roberts Edge Detection Operator*. We assume that *f*(*x*, *y*) represents a two-dimensional image, and *G*(*x*, *y*) is the gradient of the image, then we have:

(8) $$\begin{array}{c} G\left(x,y\right)={\left[f_{x}^{\prime },f_{y}^{\prime }\right]}^{T}={\left[\frac{\partial f}{\partial x},\frac{\partial f}{\partial y}\right]}^{T}. \end{array}$$

For a two-dimensional digital image, it can be represented by differential, as follows:

(9) $$\begin{array}{c} \nabla f_{x}=f\left[i+1,j\right]-f\left[i,j\right],\\ \nabla f_{y}=f\left[i,j+1\right]-f\left[i,j\right]. \end{array}$$

Among them, (*i*, *j*) represents the coordinates of the pixels in the image.

The Roberts edge detection operator is the earliest operator that uses the difference operator to detect edges. The mathematical expression of the algorithm is as follows:

(10) $$\begin{array}{c} \nabla f\left[i,j\right]\neq \left|G_{x}\right|+\left|G_{y}\right|. \end{array}$$

That is:

(11) $$\begin{array}{c} \nabla f\left[i,j\right]=\left|f\left[i+1,i\right]-f\left[i,j\right]\right|+\left|f\left[i,j+1\right]-f\left[i,j\right]\right|. \end{array}$$

The convolution templates *G*_*x*_ and *G*_*y*_ are, respectively as follows:

(12) $$\begin{array}{c} G_{x}=\left[\begin{array}{cc} 1 & 0\\ 0 & -1 \end{array}\right],\\ G_{y}=\left[\begin{array}{cc} 0 & 1\\ -1 & 0 \end{array}\right]. \end{array}$$

It can be seen from the convolution template that the Roberts edge detection operator uses the neighborhood of the current position pixel 2 × 2. Therefore, the algorithm has a small amount of calculation, but it is also very sensitive to noise, so this operator is often used in occasions with less noise.

*(2) Sobel Edge Detection Operator*. The Sobel edge detection operator is also a first-order differential edge detection operator like the Roberts edge detection operator, and the convolution template of the Sobel operator is 3 × 3. (*i*, *j*) is the center of the matrix, then the partial derivative at point (*i*, *j*) is as follows:

(13) $$\begin{array}{c} \nabla f_{x}=\left(a_{2}+ca_{4}+a_{7}\right)-\left(a_{0}+ca_{3}+a_{5}\right),\\ \nabla f_{y}=\left(a_{0}+ca_{1}+a_{2}\right)-\left(a_{5}+ca_{6}+a_{7}\right). \end{array}$$

Among them, when *c* = 2, the model is the Sobel edge detection operator, and when *c* = 1, the model is the Prewitt edge detection operator, and the convolution template is as follows:

*(3) Kirsch Edge Detection Operator*. Different from the convolution kernels of the first two edge detection operators, the Kirsch edge detection operator consists of 8 convolution kernels. When detecting the edge of the image, each convolution kernel represents a direction, and each pixel must be convolved with these 8 convolution kernels. Different convolution kernels represent the maximum response in this direction, and the 8 maximum values are taken as the output of the edge.

*(4) Canny Edge Detection Operator*. The actual image signal usually contains noise, and both noise and edge appear as high-frequency signals in the image spectrum. If the previous algorithms are used to detect a large amount of noise in the image as false edges, the Canny edge detection operator first smoothes the image to filter out the noise and then detects the edges, which can avoid the detection of noise false edges. We assume that *h*(*x*, *y*) is a Gaussian filter function, and the smoothed image is *g*(*x*, *y*), then there are:

(14) $$\begin{array}{c} \nabla g\left(x,y\right)=\nabla \left(f\left(x,y\right)⊗h\left(x,y\right)\right)=f\left(x,y\right)⊗\nabla h\left(x,y\right). \end{array}$$

After the image is processed by Gaussian filtering, the edges will be blurred, so the detected edges will be thicker. The wide edges are thinned by nonmaximum suppression (NMS) method on the gradient magnitude, and finally the edges are connected by a double-threshold method.

*(5) Traditional Arts and Crafts Image Edge Detection Operator*. The first few operators are all first-order differential edge detection operators, and edge detection is performed by solving the extreme value of the first-order differential of the image. This calculation method may result in nonunique detection of edge points. The traditional arts and crafts image edge detection operator is a second-order differential edge detection operator, and the edge point can be determined by calculating the zero point of the second-order differential. Therefore, the second-order differential edge detection operator is more accurate than the first-order differential edge detection operator, but the disadvantage is that the second-order differential edge detection operator is susceptible to noise. Therefore, the traditional arts and crafts image edge detection operator is to first perform Gaussian filtering on the original image, and then perform second-order differentiation, which will increase the antinoise ability of the operator. The model of the Laplacian operator is as follows:

(15) $$\begin{array}{c} \nabla^{2}f\left(x,y\right)=\frac{\partial^{2}}{\partial x^{2}}f\left(x,y\right)+\frac{\partial^{2}}{\partial y^{2}}f\left(x,y\right). \end{array}$$

The discrete form is as follows:

(16) $$\begin{array}{c} \nabla^{2}f\left[i,j\right]=f\left[i+1,j\right]+f\left[i-1,j\right]+f\left[i,j+1\right]+f\left[i,j-1\right]-4f\left[i,j\right]. \end{array}$$

We assume that *h*(*x*, *y*) is a Gaussian filter function, then the mathematical model of the traditional arts and crafts image edge detection operator is as follows:

(17) $$\begin{array}{c} \nabla^{2}g\left(x,y\right)=\nabla^{2}\left[f\left(x,y\right)⊗h\left(x,y\right)\right]=0. \end{array}$$

According to the nature of the convolution operation, there are

(18) $$\begin{array}{c} \nabla^{2}g\left(x,y\right)=f\left(x,y\right)⊗\nabla^{2}h\left(x,y\right). \end{array}$$

Among them, there are

(19) $$\begin{array}{c} \nabla^{2}h\left(x,y\right)=\frac{1}{2\pi \delta^{4}}\left(\frac{x^{2}+y^{2}}{\delta^{2}}-2\right)e^{-x^{2}+y^{2}/2\delta^{2}}. \end{array}$$

Figure 5 shows the traditional arts and crafts image operator and its spectrogram. The function has a zero at *t*=±*δ*, and it can be proved that the integral of the function is zero over the entire interval. Owing to the smoothness of ∇^2^*h*(*x*, *y*), the traditional arts and crafts image operator can accurately obtain the position of the edge when the noise is large or the edge is not clear.

*(6) Improved Gabor Edge Detection Operator*. In the research field of image processing, the Gabor kernel function model is often used for edge description, extraction, and detection of textures. The characteristics of the Gabor model in frequency and direction are very close to the human visual system. The complex model of the two-dimensional Gabor filter is as follows:

(20) $$\begin{array}{c} g\left(x,y,\lambda ,\theta ,\psi ,\sigma ,\gamma \right)=\exp\left(-\frac{x_{1}^{2}+\gamma^{2}y_{1}^{2}}{2\sigma^{2}}\right)\exp\left(i\left(2\Pi \frac{x_{1}}{\lambda }+\psi \right)\right). \end{array}$$

The real part expression is as follows:

(21) $$\begin{array}{c} g\left(x,y,\lambda ,\theta ,\psi ,\sigma ,\gamma \right)=\exp\left(-\frac{x_{1}^{2}+\gamma^{2}y_{1}^{2}}{2\sigma^{2}}\right)\cos\left(2\Pi \frac{x_{1}}{\lambda }+\psi \right). \end{array}$$

The imaginary part expression is as follows:

(22) $$\begin{array}{c} g\left(x,y,\lambda ,\theta ,\psi ,\sigma ,\gamma \right)=\exp\left(-\frac{x_{1}^{2}+\gamma^{2}y_{1}^{2}}{2\sigma^{2}}\right)\sin\left(2\Pi \frac{x_{1}}{\lambda }+\psi \right). \end{array}$$

Among them, there are:

(23) $$\begin{array}{c} \left\{\begin{array}{c} x_{1}=x\;\cos\;\theta +y\;\sin\;\theta ,\\ y_{1}=-x\;\sin\;\theta +y\;\cos\;\theta . \end{array}\right. \end{array}$$

An improved Gabor filter model is proposed. The improved Gabor function model not only has good characteristics in direction and scale but also has good curve recognition ability. The two improved Gabor models are as follows:

(a) Gabor function model based on Taylor series is as follows
  (24) $$\begin{array}{c} \left\{\begin{array}{c} x_{1}=x\;\cos\;\theta +y\;\sin\;\theta +\sum_{i=1}^{n}m_{i}{\left(\alpha x\;\sin\;\theta +\beta y\;\cos\;\theta \right)}^{i+1},\\ y_{1}=-x\;\sin\;\theta +y\;\cos\;\theta . \end{array}\right. \end{array}$$
First, the concept of Taylor series is introduced here, so from formula (23), it can be seen that the relationship between *x*_1_ and *y*_1_ satisfies the definition of Taylor's formula, and *x*_1_ and *y*_1_ no longer exhibit a linear relationship due to the latter nonlinear factor ∑_*i*=1_^*n*^*m*_*i*_(*αx*  sin  *θ*+*βy*  cos  *θ*)^*i*+1^. Taylor's formula is as follows:
  (25) $$\begin{array}{c} f\left(x\right)=\frac{f\left(a_{0}\right)}{0!}+\frac{f{\left(a_{0}\right)}^{\prime }}{1!}\left(x-a_{0}\right)+\frac{f{\left(a_{0}\right)}^{\prime \prime }}{2!}{\left(x-a_{0}\right)}^{2}+\cdots \frac{f^{\left(n\right)}\left(a_{0}\right)}{n!}{\left(x-a_{0}\right)}^{n}+R\left(x\right). \end{array}$$
It can be seen from the aforementioned formula that any smooth curve function analytical formula can be expanded by Taylor formula. Usually in formula (24), *α* takes −1, *β* takes 1, *m*_1_ is the parameter for adjusting the basic trend of the curvature, and *m*_2_ is the parameter for adjusting the details of the curvature. By adjusting *m*_1_ and *m*_2_, the improved Gabor model can detect the ridges of the curved part of the fingerprint well.
(b) Improvement of Gabor function model based on Fourier series is as follows:
  (26) $$\begin{array}{c} \left\{\begin{array}{c} x_{1}=x\;\cos\;\theta +y\;\sin\;\theta +\sum_{k=1}^{n}m_{k}\left(-x\;\sin\;k\theta +y\;\cos\;k\theta \right),\\ y_{1}=-x\;\sin\;\theta +y\;\cos\;\theta . \end{array}\right. \end{array}$$
First, the Fourier series is introduced. Therefore, it can be seen from formula (27) that the relationship between *x*_1_ and *y*_1_ satisfies the definition of Taylor's formula, and from the nonlinear factor behind formula (24), it can be seen that *x*_1_ and *y*_1_ no longer exhibit a linear relationship, and the Fourier series is as follows:
  (27) $$\begin{array}{c} f\left(t\right)=A_{0}+\sum_{n=1}^{\infty }\left(A_{n}\sin\;n\omega t+B_{n}\cos\;n\omega t\right). \end{array}$$
Among them, there are:
  (28) $$\begin{array}{c} \left\{\begin{array}{c} A_{0}=\frac{1}{\pi }\int_{-\pi }^{\pi }f\left(t\right)\text{d}t,\\ A_{n}=\frac{1}{\pi }\int_{-\pi }^{\pi }f\left(t\right)\cos\;nt\text{d}t,\\ B_{n}=\frac{1}{\pi }\int_{-\pi }^{\pi }f\left(t\right)\sin\;nt\text{d}t. \end{array}\right. \end{array}$$

It can be seen that the Fourier series expansion can be used for any analytic expression of the smooth curve function that conforms to the Dirichlet constraint. Usually, *s* is taken. By adjusting the value of *k*, the improved Gabor filter can detect the edge of the curved part of the image well.

For a two-dimensional discrete digital image, according to the definition of Taylor series, the neighborhood pixels of any pixel *x*_0_ and *y*_0_ can be expressed as the expanded form of two-dimensional Taylor series. We assume that the Gaussian kernel function is *h*(*x*, *y*), and the result of convolving the image *f*(*x*, *y*) and *h*(*x*, *y*) is *g*(*x*, *y*), then the partial derivative of the Gaussian kernel function *h*(*x*, *y*) is as follows:

(29) $$\begin{array}{c} \left\{\begin{array}{c} h_{x}\left(x,y\right)=h^{\prime }\left(x\right)h\left(y\right),\\ h_{y}\left(x,y\right)=h^{\prime }\left(y\right)h\left(x\right),\\ h_{xx}\left(x,y\right)=h^{\prime \prime }\left(x\right)h\left(y\right),\\ h_{xy}\left(x,y\right)=h^{\prime }\left(x\right)h^{\prime }\left(y\right),\\ h_{yy}\left(x,y\right)=h^{\prime \prime }\left(y\right)h\left(x\right). \end{array}\right. \end{array}$$

Then, the two-dimensional quadratic Taylor expansion of the image at (*x*_0_, *y*_0_) is as follows:

(30) $$\begin{array}{c} f\left(x,y\right)=g\left(x_{0},y_{0}\right)+\left(x-x_{0}\right)\left(y-y_{0}\right)\left(\begin{array}{c} g_{x}\left(x_{0},y_{0}\right)\\ g_{y}\left(x_{0},y_{0}\right) \end{array}\right)\\ +\frac{1}{2}\left[\left(x-x_{0}\right)\left(y-y_{0}\right)\right]\left[\begin{array}{cc} g_{xx}\left(x_{0},y_{0}\right) & g_{xy}\left(x_{0},y_{0}\right)\\ g_{yx}\left(x_{0},y_{0}\right) & g_{yy}\left(x_{0},y_{0}\right) \end{array}\right]\left[\begin{array}{c} \left(x-x_{0}\right)\\ \left(y-y_{0}\right) \end{array}\right]. \end{array}$$

We assume that the edge normal vector is *n*(*x*, *y*)=(*n*_*x*_, *n*_*y*_). In a two-dimensional image, the point where the first-order directional derivative is zero or the extreme point of the second-order directional derivative is the center point of the edge. Therefore, if the normal direction *n*(*x*, *y*) of the image edge is known, the aforementioned formula can be expressed as follows:

(31) $$\begin{array}{c} f\left(\left(tn_{x}+x_{0}\right),\left({\mathrm{tn}}_{y}+y_{0}\right)\right)=g\left(x_{0},y_{0}\right)+tn_{x}g_{x}\left(x_{0},y_{0}\right)+{\mathrm{tn}}_{y}g_{y}\left(x_{0},y_{0}\right)\\ +\frac{1}{2}t^{2}n_{x}^{2}g_{xx}\left(x_{0},y_{0}\right)+\frac{1}{2}t^{2}n_{y}^{2}g_{yy}\left(x_{0},y_{0}\right)+t^{2}n_{x}n_{y}g_{xy}\left(x_{0},y_{0}\right). \end{array}$$

For the edge of the image, cross ∂/∂*tf*((*tn*_*x*_+*x*_0_), (*tn*_*y*_+*y*_0_))=0, we get

(32) $$\begin{array}{c} t=\frac{n_{x}g_{x}+n_{y}g_{y}}{n_{x}^{2}g_{xx}+2n_{x}n_{y}g_{xy}+n_{y}^{2}g_{yy}}. \end{array}$$

The algorithm substitutes *t* into ((*tn*_*x*_+*x*_0_), (*tn*_*y*_+*y*_0_)), which is the position of the extreme point pixel of the image gray level. If (*tn*_*x*_, *tn*_*y*_) ∈ [−1/2, 1/2] × [−1/2, 1/2], the extreme point is located at the center point of the edge, and the precision of this point is subpixel-level smaller than the pixel. The edge normal vector (*n*_*x*_, *n*_*y*_) and the second-order differential of the direction are obtained by the Hessian matrix *H*(*x*, *y*) of the two-dimensional image, and its expression is as follows:

(33) $$\begin{array}{c} H\left(x,y\right)=\left[\begin{array}{cc} g_{xx} & g_{xy}\\ g_{yx} & g_{yy} \end{array}\right]. \end{array}$$

It has been proved that the extreme point of the second-order differential of the image function is the two eigenvalues of the Hessian matrix, and the direction of the extreme value is the eigenvector of the Hessian matrix. Therefore, the edge normal vector (*n*_*x*_, *n*_*y*_) and its second derivative can be obtained by obtaining the extreme value of the Hessian matrix and the corresponding eigenvector. The normal vector (*n*_*x*_, *n*_*y*_) of the image edge and the position of the second-order directional derivative subpixel ((*tn*_*x*_+*x*_0_), (*tn*_*y*_+*y*_0_)) of the image edge are obtained through the Hessian matrix. The algorithm starts from the pixels of the image edge intensity and adds appropriate neighborhood points to form a line, the algorithm determines whether the neighborhood point should be added to the edge line by the difference between the distance and the angle between the selected neighborhood point and the current edge center point, that is, we assume that *d* is the distance difference between the selected neighborhood point and the current edge center point, and *θ*(*θ* ∈ [0, *π*/2]) is the angle difference between the selected neighborhood point and the current edge center point. Then, the neighborhood points when *d*+*θ* is the minimum value can be added to the edge line, and the purpose of edge detection based on subpixels is finally achieved through the connection of the edge.

In this paper, the feature alignment method based on image contour moments is used to align the two images. The flow chart of the algorithm is shown in Figure 6. First, the algorithm needs to perform image preprocessing, edge contour extraction, and tracking merging on the template image and the image to be matched, respectively. The flow chart of the alignment method based on the image contour moment is shown in Figure 6.

The algorithm mainly includes two points: extraction of contour moment feature, parameter calculation, and affine transformation. The most important thing is that the extraction of contour moment features and parameter calculation are divided into two steps:

*(1) Calculate the Centroid of the Contour Image*. We assume a binary image is *f*(*x*, *y*), the image centroid position is (*x*_*c*_, *y*_*c*_), then the mn-order center distance of the image is expressed as follows:

(34) $$\begin{array}{c} M_{mn}=\sum_{i=0}^{m}\sum_{j=0}^{n}f\left(x_{i},y_{j}\right){\left(x_{i}-x_{c}\right)}^{m}{\left(y_{j}-y_{c}\right)}^{n}. \end{array}$$

Based on the principle that the centroids of the images should be as close as possible to the complete registration of the two images, the translation amount *T* between the image to be matched and the template image can be determined by the geometric centroids of the two images. Since *f*(*x*, *y*) is a binarized contour image, its centroid can be expressed as follows:

(35) $$\begin{array}{c} x_{c}=\frac{M_{10}}{M_{00}}=\frac{\sum_{i=0}^{m}\sum_{j=0}^{n}x_{i}f\left(x_{i},y_{i}\right)}{\sum_{i=0}^{m}\sum_{j=0}^{n}f\left(x_{i},y_{i}\right)},\\ y_{c}=\frac{M_{10}}{M_{00}}=\frac{\sum_{i=0}^{m}\sum_{j=0}^{n}y_{i}f\left(x_{i},y_{i}\right)}{\sum_{i=0}^{m}\sum_{j=0}^{n}f\left(x_{i},y_{i}\right)}. \end{array}$$

*(2) Calculate the Main Axis Angle of the Contour Image*. We assume that the angle between the main axis of the contour image and the vertical axis is *θ*, and there are

(36) $$\begin{array}{c} \theta =\frac{1}{2}\arctan\left(\frac{2M_{11}}{M_{20}-M_{02}}\right). \end{array}$$

Finally, the algorithm can complete the image alignment through the translation amount *T* and the included angle.

Figure 7 shows the relationship between the gray value difference and the processed gray value in the improved algorithm. After comparing the detection results of these two methods, it is found that the algorithm in this paper is more suitable for the detection requirements of the system and the enterprise.

## 4. An Intelligent Analysis System for Traditional Arts and Crafts Based on Digital technology: Taking the Guangdong-Hong Kong-Macao Greater Bay Area as the Observation Center

In the third part, an intelligent analysis system of traditional arts and crafts based on digital technology is constructed. Next, this article takes the Guangdong-Hong Kong-Macao Greater Bay Area as the observation center, and collects the traditional arts and crafts works in the Guangdong-Hong Kong-Macao Greater Bay Area for research. This paper conducts experimental analysis through multiple groups of traditional arts and crafts works in the Greater Bay Area of Macao, and verifies the effect of the traditional arts and crafts intelligent analysis system based on digital technology proposed in this paper and counts the effect of the system in the intelligent analysis of arts and crafts in the Guangdong-Hong Kong-Macao Greater Bay Area. The results are shown in Tables 1 and 2. Among them, Table 1 is the digital analysis effect of traditional arts and crafts in Guangdong-Hong Kong-Macao Greater Bay Area, and Table 2 is the intelligent analysis effect of arts and crafts of traditional arts and crafts intelligent analysis system in Guangdong-Hong Kong-Macao Greater Bay Area.

From the aforementioned research, it can be seen that the intelligent analysis system of traditional arts and crafts based on digital technology proposed in this paper is very effective. With the support of this system, the intelligent analysis of traditional arts and crafts in Guangdong-Hong Kong-Macao Greater Bay Area can be carried out efficiently.

## 5. Conclusion

In the development of traditional arts and crafts, it is necessary to actively absorb other forms of artistic expression. The development and design of traditional arts and crafts is a direct manifestation of the spread of traditional culture. Moreover, it clearly shows the development trend of traditional Chinese culture. The cultures of different regions influence and promote each other, and the characteristics of folk customs have gradually become the main driving force for the development of cultural integration. At the same time, traditional arts and crafts can better reflect modern life, truly give full play to the functions of traditional arts and crafts, so that more people can embrace traditional arts and crafts and inject new vitality into development. This paper analyzes traditional arts and crafts combined with digital technology, builds an intelligent analysis system, and improves the digital processing effect of traditional arts and crafts. The experimental research shows that the traditional arts and crafts intelligent analysis system based on digital technology proposed in this paper has a very good effect. With the support of this system, the intelligent analysis of traditional arts and crafts in the Guangdong-Hong Kong-Macao Greater Bay Area can be carried out efficiently.

## Figures and Tables

**Figure 1:** Step (1).

**Figure 2:** Step (2).

**Figure 3:** Image enhancement comparison chart: (a) original image, (b) processing diagram of histogram equalization algorithm, and (c) the graph processed by the algorithm in this paper.

**Figure 4:** OTSU threshold segmentation.

**Figure 5:** Spectrogram of traditional arts and crafts image operator.

**Figure 6:** Flow chart of image alignment.

**Figure 7:** Improved algorithm (gray-difference).

**Table 1:** The digital analysis effect of the traditional arts and crafts intelligent analysis system in the Guangdong-Hong Kong-Macao Greater Bay Area.

Number	Work analysis	Number	Work analysis	Number	Work analysis
1	79.78	19	83.34	37	81.31
2	76.79	20	81.28	38	77.91
3	82.87	21	76.11	39	81.14
4	74.08	22	80.89	40	73.21
5	75.92	23	83.36	41	73.61
6	79.37	24	74.20	42	83.37
7	83.30	25	78.72	43	72.83
8	72.16	26	76.58	44	78.48
9	72.82	27	73.70	45	81.33
10	76.64	28	72.35	46	82.14
11	75.54	29	72.38	47	83.60
12	77.02	30	81.76	48	73.17
13	72.57	31	77.72	49	83.50
14	74.99	32	78.25	50	75.20
15	74.13	33	79.24	51	82.12
16	76.91	34	79.30	52	77.94
17	83.08	35	71.82	53	71.03
18	77.50	36	81.19	54	74.51

**Table 2:** The intelligent analysis effect of arts and crafts of the traditional arts and crafts intelligent analysis system in Guangdong-Hong Kong-Macao Greater Bay Area.

Number	Art analysis	Number	Art analysis	Number	Art analysis
1	74.42	19	80.73	37	77.95
2	85.44	20	83.90	38	80.68
3	80.79	21	84.21	39	76.48
4	73.93	22	75.19	40	75.86
5	73.13	23	73.55	41	82.04
6	77.60	24	83.45	42	75.06
7	86.24	25	87.48	43	86.36
8	74.49	26	85.67	44	86.76
9	74.32	27	78.28	45	82.58
10	84.27	28	73.04	46	87.89
11	79.55	29	86.32	47	75.60
12	87.50	30	74.80	48	76.17
13	73.77	31	86.24	49	77.42
14	74.34	32	85.80	50	82.00
15	86.72	33	80.76	51	84.39
16	78.91	34	76.48	52	86.13
17	84.14	35	75.07	53	86.74
18	84.81	36	87.38	54	75.33

## Data Availability

The labeled data set used to support the findings of this study is available from the corresponding author upon request.
